# ‘I wanted to enjoy our marriage first… but I got pregnant right away’: a qualitative study of family planning understandings and decisions of women in urban Yogyakarta, Indonesia

**DOI:** 10.1186/s12884-018-1991-y

**Published:** 2018-08-30

**Authors:** Belinda Rina Marie Spagnoletti, Linda Rae Bennett, Michelle Kermode, Siswanto Agus Wilopo

**Affiliations:** 1 The Nossal Institute for Global Health, Melbourne School of Population and Global Health, Faculty of Medicine, Dentistry and Health Sciences, The University of Melbourne, 333 Exhibition Street, Melbourne, VIC 3000 Australia; 2 Center for Reproductive Health, Faculty of Medicine, Gadjah Mada University, Jalan Farmako Sekip Utara, Yogyakarta, 55281 Indonesia; 3 Department of Biostatistics, Epidemiology and Public Health, Faculty of Medicine, Gadjah Mada University, Jalan Farmako Sekip Utara, Yogyakarta, 55281 Indonesia

**Keywords:** Family planning, Contraception, Postpartum health, Reproductive health, Indonesia, Reproductive agency, Quality of care, Interpersonal relationships, Societal norms, Family planning providers

## Abstract

**Background:**

Despite several decades of investment into family planning and maternal health systems strengthening, Indonesia’s maternal mortality ratio remains among the highest in Southeast Asia. Among postpartum women unmet need for family planning is greater than at any other time, thus there is great potential to improve the reproductive health outcomes of Indonesian women through enhanced postpartum family planning access. This article explores the socially embedded nature of family planning choices in the Indonesian context, drawing on the experiences of a sample of urban dwelling and predominantly middle class women.

**Methods:**

This was an ethnographic study which explored the reproductive experiences of women residing in Yogyakarta City, and Sleman and Bantul regencies. Fieldwork was undertaken over 18 months from September 2014 to March 2016. This article draws on 31 in-depth interviews (IDIs) conducted with 20 women aged 21 to 38 years who had given birth less than two years prior.

**Results:**

Though there was great variance across women’s reproductive trajectories, the majority had limited understandings of family planning, especially in relation to contraception. Societal norms pertaining to women’s fertility and reproduction underpinned women’s desires to become pregnant soon after marriage. Normative ideals concerning family size and the composition of families underpinned women’s desires for a maximum of two to three children, with at least one child of each sex. Negotiations concerning timing of pregnancies and family size occurred within spousal relationships. The majority of women were using some form of fertility control to prevent or space pregnancies, with method choice decisions often informed by family members, friends and family planning providers. Quality of care among family planning providers was often lacking, perpetuating misinformation, and women’s choices were not always respected.

**Conclusions:**

Our analysis reveals the socially embedded nature of women’s postpartum family planning understandings and choices, and the ways in which social and relational factors sometimes constrain and at other times support women’s reproductive agency. We identify key areas for health sector reform to enhance women’s understandings of postpartum family planning and improve family planning quality of care.

## Background

Since the 1980s the Government of Indonesia (GoI) has committed to a range of health system strengthening measures aimed at improving maternal health [1, 2]. Yet the country’s maternal mortality rate (MMR) – estimated to be between 126 to 359 deaths per 100,000 live births – remains well above the regional average of 110 [3, 4].^1^ Indonesia’s MMR is also much higher than other Southeast Asian states that have experienced similarly rapid economic growth and urbanisation, most notably Thailand (MMR = 20), Malaysia (MMR = 40) and Vietnam (MMR = 54) [4]. Postpartum haemorrhage, preeclampsia and eclampsia are the leading causes of maternal deaths and near-miss deaths in Indonesia [1]. Though home births without the aid of trained birth attendants remain commonplace in certain areas [5, 6], almost half of all maternal deaths in Indonesia occur at district or provincial hospitals [1]. Delayed access to medical treatment can result in the escalation of treatable maternal conditions to fatalities. Recent studies reveal that delayed medical attention is a consequence of factors related to poverty, geography, or the absence of quality maternal health care [1, 7, 8]. Most disconcerting is the fact that while maternal health has been a central pillar of the GoI’s framing of reproductive health, and after more than three decades of health systems strengthening in the area, outcomes for Indonesian women remain poor and among the worst in Southeast Asia.

Family planning, embodied by the national family planning program, is another key pillar of the GoI’s delineation of reproductive health. Aimed at controlling population growth through the provision of contraception to Indonesian women and couples, family planning has been strongly promoted by the GoI since the 1970s ahead of other areas of reproductive health [9]. Fertility control achieved via family planning can markedly improve both maternal and child health [10–13]. This is particularly the case in lower income settings, such as Indonesia, where death and illness associated with pregnancy and deliveries are more commonplace, and is the basis for growing calls by public health advocates to promote postpartum family planning [10, 14]. Paradoxically, unmet need for family planning during the first year following delivery is greater than at any other time, despite the fact that most women seek to delay or prevent future pregnancies during the extended postpartum period [14, 15]. Postpartum contraception helps couples to space and prevent future pregnancies safely [10]. Unintended pregnancies are more likely to negatively impact on the health, social and economic circumstances of women and their families than planned pregnancies [16, 17]. Current World Health Organization (WHO), guidelines recommend offering women biomedical contraception – even if their menses have not resumed – before the sixth week postpartum [18]. The WHO recommends a range of contraceptive options for postpartum women, a number of which can be used immediately after delivery and while breastfeeding [19]. Of the biomedical contraceptives available in Indonesia there are a range of methods that can safely be used during the postpartum period and in conjunction with breastfeeding. At any time immediately following childbirth and during the first six weeks (and beyond) postpartum contraceptive implants, progestogen-only pills (POP) and condoms may be used [19]. Additionally, after six weeks progestogen-only injectable contraceptives can be used [19]. Copper intrauterine devices (IUDs), which are the only variant of IUDs available in Indonesia, can be inserted within the first 48 h postpartum or any time after the first four weeks [19].

Recent Indonesian Demographic and Health Surveys (IDHSs) have revealed that the fertility and family planning behaviours of women in Yogyakarta, the field site of this study, are distinctive compared with other parts of Indonesia. The total fertility rate (TFR) in Yogyakarta has remained well below the national rate of 2.6; however the TFR in the 2012 IDHS (2.1) is the highest recorded in 25 years since the 1987 IDHS [3, 20–23]. Compared to women in other parts of Java, women in Yogyakarta experience the highest rates of postpartum amenorrhea, postpartum abstinence and postpartum insusceptibility [3]. In comparison with the general population, women in Yogyakarta also wish to control their fertility after they have achieved a family size of two or three children. Of women with two children, 87% want no additional children compared with 60% nationally; and of those with three children, 97% want no additional children compared with 80% nationally [3]. Yogyakarta also has the second highest prevalence of traditional contraceptive use among married women, with 10.3% of women relying on the withdrawal and periodic abstinence methods compared with 4% of women nationally [3]. Use of the copper IUD is also more prevalent among women Yogyakarta (13.6%), compared with women nationally (3.9%) [3].

Several recent African studies have explored the contraception and fertility preferences of postpartum women [24, 25]. These studies highlight the utility of qualitative explorations into women’s reproductive lives and subjectivities beyond the narrow definition of unmet need for family planning, which, according to Rusibamayila and colleagues [25], ‘inadequately capture and convey the multilevel factors that institutionalise preferences and influence action, generating the gap between reported intentions and enacted fertility behaviour’. An emerging body of literature focuses on key interpersonal relationships influencing the reproductive health decisions of women in South Asia [26–28] and in Africa [29–31]. These studies reveal women’s complex interactions with their husbands, other family and community members, and the health system, which inform their reproductive health understandings and choices. The analytical thread linking these studies is their conceptualisations of women’s reproductive agency to make decisions that influence their reproductive health, notwithstanding the limitations placed on their autonomy. Mumtaz and Salway [17] have critiqued the relevance of the concept of autonomy as it applies to the reproductive health of women living in lower income countries. They argue that to assume women’s use of reproductive healthcare constitutes independent and autonomous decision making overlooks the interdependent kin relationships in which their identities are deeply embedded [17]. We concur with Mumtaz and Salway’s perspective in the Indonesian context, and consider the notion of reproductive agency to be more nuanced and suitable for our analysis than the notion of autonomous decision making. Reproductive agency has been aptly defined by Unnithan-Kumar [32] as ‘the ideas, actions, thinking and planning in the domain of human reproduction by women and men who engage in reproductive activities and seek healthcare services’.

Recent research in Indonesia has considered ways in which women’s interpersonal relationships, alongside geographical, cultural and economic factors, influence their uptake of antenatal and postnatal care [5, 33–37]. With the exception of a recent quantitative analysis by Wilopo and colleagues [38], postpartum family planning remains underexplored in the Indonesian context, and this is a key contribution of this study. In addition, qualitative studies on women’s reproductive health in Indonesia have tended to focus on the experiences of less affluent women [5, 7, 33, 37, 39–41]. Enquiry into the reproductive lives of middle class Indonesian women has been rather more limited, with the exception of Bennett’s [42, 43] recent work on infertility. This study thus contributes to an emerging body of research that considers the reproductive health needs of Indonesia’s growing middle class population. Aligned with studies in other lower income settings referred to above, this article focuses on the normative social expectations and relational factors – including interactions with the health system – that influence the understandings and decisions of postpartum women in relation to family planning. This study explored the reproductive narratives of women who had recently given birth in urban Yogyakarta. Interviews traced women’s understandings of family planning and the values that they attributed to family planning.

## Methods

Findings from the first author’s doctoral fieldwork, conducted over an 18-month period from September 2014 to March 2016, inform this analysis. The study employed an ethnographic approach to explore the family planning understandings and experiences of middle class women residing in urban Yogyakarta, Indonesia (see Table 1). The definition of the postpartum period that we adopt in this study extends to the first year following a woman’s delivery, often referred to as the extended postpartum period [14]. Ethnographic methods have been well tested by a lineage of researchers in Southeast and South Asia in their investigations of women’s reproductive and sexual health and rights, including Bennett [39, 40, 43], Chakraborty [44], Parker [45, 46] and Raman [27, 28, 47]. The Center for Reproductive Health at Gadjah Mada University provided an institutional base and the Center’s Director, SAW, sponsored BRS to obtain the required foreign research permit from the Indonesian Ministry of Research and Technology. Findings from this study on the other key research themes have been published elsewhere. These themes have included breastfeeding health promotion and related embodiment by participants [48]; and participants’ experiences of balancing their reproductive and productive lives [49].

**Table 1:** Family planning themes explored during in-depth interviews

Family planning understandings, intentions and experiences	
Intended family size	
Planned and actual spacing between pregnancies	
Contraceptive histories	
Fertility problems	
Resumption of intimate relationship postpartum	
Postpartum family planning, including fertility control plans or contraception use	

### Field site

Yogyakarta is a special administrative region physically surrounded by the province of Central Java. It is Indonesia’s second smallest province, spanning just 3,133km^2^. Approximately 3.66 million people reside in Yogyakarta, making it the fourth most densely populated province in Indonesia. Almost three-quarters of the population is urban-dwelling. Islam is the predominant religion, followed by Catholicism and other schools of Christianity.

### Study design

Multiple qualitative methods were used. These methods included in-depth interviews (IDIs), focus group discussions, semi-structured interviews, and participant observation. Consistent with an ethnographic approach, data collection and analysis were iterative and undertaken across several stages. The utility of an ethnographic approach is that it allows the researcher to move closer to an in-depth understanding of the research phenomena. Multiple non-probability sampling techniques were employed as described below. Participants were recruited from the capital city, Kota Yogyakarta, and the two most urbanised regencies, Sleman and Bantul. Participant recruitment was facilitated by the Department of Health, Kota Yogyakarta and the Indonesian Breastfeeding Mothers’ Association (AIMI). The total sample size was 39 participants, including 20 women who participated in IDIs. IDI participants are the core group of informants whose experiences this study sought to understand, and their narratives provide the basis for analysis in this article.

### Sampling and recruitment

A common sampling strategy in ethnographic research is to rely on multiple non-probability approaches to derive a sample [50]. In this study the sample was recruited in three stages: an initial sample was recruited; followed by a theoretical sample; and in the third stage a deviant case sample was recruited [50–52]. A homogeneous sample of women, who had given birth within the last two years, aged between 20 to 40 years and living in urban Yogyakarta, was initially sought. Following preliminary data analysis undertaken by BRS with input from LRB, the sampling parameters were refined and, in addition to the initial sampling frame, a majority of Muslim women, and women who had ever breastfed, were sought. Following further analysis by BRS with input from LRB, a deviant case sample of women who had experienced challenges in breastfeeding was sought. The total sample size was informed by the ongoing analysis of participants’ narratives that occurred during the data collection phase, with IDI recruitment ceasing once data saturation was achieved. Participants were introduced to BRS through various means: five were referred by AIMI; three were recruited at AIMI events; four were recruited at a public primary health clinic; and eight were recruited via snowballing. With the exception of one participant recruited by her neighbour through whom her interview was arranged, all of the key informants received an open invitation from BRS to participate in the study. This necessitated participants to confirm their involvement in the study and thus avoid any possibility of compulsion.

### Data collection

#### In-depth interviews

The IDI guide was piloted by BRS with two women who had similar characteristics to the women the study was seeking to recruit. These pilot exercises were important to identify shortcomings in the interview guide, as well as clarify local, non-biomedical language related to the research topic. All interviews were conducted by BRS using Indonesian language primarily.^2^ IDIs were designed to gain deep understandings of informants’ perceptions and experiences in relation to their reproductive lives, including the themes in relation to family planning outlined in Table 1. Interviewing commenced in April 2015 and concluded in March 2016, during which time 20 women who had recently given birth participated in a total of 31 interviews. Rapport building was integral to relationships with participants [50]. Interview timing and location was at the discretion of participants, and the majority were held in their homes or workplaces. Participant’s children were often present, and occasionally their domestic workers, husbands, other family members or colleagues were present. Eleven women participated in a single interview, seven women participated in two interviews and two women participated in three interviews. Due to the interviews being guided by participants’ reproductive narratives, the need for BRS to build rapport with participants, the lengthier duration of first interviews, and requests for follow-up by some participants, multiple interviews were at times necessary. Three women requested that their interviews not be audio recorded, so extensive notes were taken. Interviews lasted between 23 min to 2 h and 47 min. The median duration was 1 h and 46 min. Verbatim transcripts of the audio recorded interviews were prepared by local research assistants. Participants were recompensed Rp. 50,000 (approximately USD $3.80) for their time or given a gift of similar monetary value, as is customary in this setting.

#### Participant characteristics

Participants were aged between 21 to 38 years and all had given birth within the prior two years. Eight of the women were primiparous and 12 were multiparous. All but three were both Muslim and Javanese (i.e. originating from Yogyakarta, Central or East Java). All had completed at least senior high school-level education, and 14 had attained post-secondary or tertiary qualifications. With the exception of two participants, all were either engaged in the formal work sector, self-employed, or studying.

### Ethics

Ethical clearance was obtained from both the Human Research Ethics Committee of the University of Melbourne (Australia) and the Ethics Committee of the Faculty of Medicine of Gadjah Mada University (Indonesia). To maintain ethical boundaries during recruitment, none of the participants met by BRS at AIMI events or at the primary health clinic were interviewed on the day they met. Informal written consent (in the form of text messages or WhatsApp messages) to participate in an interview was initially obtained by participants, and resulted in the scheduling of interviews.^3^ These text-based conversations allowed women to decide whether they wanted to participate in the study in a non-pressured context. Prior to interviews commencing all participants were provided with a plain language written description of the research and the informed consent form. All participants completed the written informed consent form prior to their participation in an interview.^4^ In the plain language written description of the research, participants were assured that their personal details would not be included in any documentation arising from the research to ensure confidentiality. They were also informed that any information generated by the research might be published, but that confidentiality would be maintained and no personal details would be divulged. They were also informed that their involvement in the research was voluntary and that withdrawal was permitted at any time and without personal consequence. In the plain language written description of the research and the informed consent form, the optional use of the audio recorder was raised, which three participants declined. In order to help protect participants’ confidentiality and identities, all selected a pseudonym to be used in place of their real name in all documentation arising from the research, including this article.

### Data analysis

Data analysis was a continuous and iterative process throughout data collection. Following each interview a modified version of Miles and Huberman’s ‘Contact Summary Form’ was completed [53]. This enabled immediate summarisation and initial analysis of the key points of discussion. The thematic content analysis and coding of transcripts was conducted by BRS with random checks undertaken by LRB (also fluent in Indonesian language). The data analysis procedure was informed by the three-stage sampling approach outlined above. At the end of the first stage of sampling the first comprehensive analysis of the data collected to that point was conducted. BRS read the IDI transcripts and Contact Summary Forms, and identified the initial categories and themes that had been generated (Table 2 below provides a snapshot of the data analysis trajectory). Informed by this analysis the interview guide was refined to both broaden and deepen the themes covered in IDIs. During the second stage of data collection BRS continued to review the new transcripts and Contact Summary Forms, identifying any additional themes that emerged, and simultaneously began coding the data and generating memos. At the conclusion of the third stage of data collection BRS re-read all of the transcripts and continued to code and interpret the results, including the consideration of rival explanations [54]. Data analysis was aided by NUDIST qualitative data analysis software (NVivo 10).

**Table 2:** Sample data analysis trajectory

Participant	Interview excerpt	Codes assigned	Key themes
Nian, 36	Perhaps if I didn’t have C-section births … I’d actually like to have a lot of children, maybe three of four … But because of my health, I think 2 is enough for now and I have to finish my studies too.	• Health limits to family size • Achieved preferred family size • Seeks to prevent future pregnancy • Balancing reproduction & production (study)	Family size Spacing pregnancies and fertility control
Fina, 31	I want 2 children and my husband agrees; we don’t want any more. The family is complete; we have a boy and a girl. Maybe if our second wasn’t a girl we would have tried again.	• Spousal agreement re number of children • Achieved preferred family size • Seeks to prevent future pregnancy • Desire for child of each sex	Family size Spacing pregnancies and fertility control
Gita, 36	If you ask me personally I already have enough … I give my breastmilk to 8 children; 3 of whom are my biological children. I would be worried I wouldn’t have the capacity to love and care for more kids than my 3 …. But of course it is ultimately up to God … and how many he gives us.	• Achieved preferred family size • Seeks to prevent future pregnancy • Religious fatalism • Demands of parenting	Family size Spacing pregnancies and fertility control
Ina, 36	My doctor recommended a sterilisation ... I asked my husband, mother and sister for advice … my sister suggested I try an IUD instead, she said that a sterilisation might decrease my hormone levels … I eventually decided to go with the IUD … it was inserted immediately after my C-section … we sometimes use condoms too, for extra safety.	• Family planning (KB)^a^ advice – KB provider • KB advice – family or friends • Concerns re KB side effects • Postpartum contraception use • Seeks to prevent future pregnancy	Spacing pregnancies and fertility control Accessing postpartum family planning
Dina, 29	I think a 4 or 5 year gap between pregnancies is ideal … my husband and I are of the view that it will be easier once our daughter is older. She’ll be able to settle by herself, be more independent… Hopefully she’ll be able to help with the baby too… it’s also about finances, when they’re older and start junior high school, senior high school…	• Desired space between pregnancies > 2 years • Seeks to delay future pregnancy • Demands of parenting • Financial cost of children	Spacing pregnancies and fertility control
Indah, 27	I didn’t use KB before my first pregnancy because it is not permitted.	• KB use constrained • Perception KB for couples with children	Family planning following marriage

^a^We have abbreviated the term ‘family planning’ to ‘KB’ as this is the term most commonly used in Indonesia

## Results

### Family planning following marriage

All participants shared the normative understanding that the purpose of marriage was to have children and that pregnancy should soon follow one’s nuptials. Thus, although biomedical contraception is legally available to all married women, it is seldom accessed by those who have not had children. Consequently none of the participants had used biomedical contraception for fertility control prior to the birth of their first child. For women who married in their late twenties and thirties this perception was amplified due to concerns that their fertility may be compromised because of their age:

I didn’t get pregnant immediately like people normally do … we were a mature age when we married, so we needed to have children right away.

Nurul, 37 (married at age 30)

However, the narratives of several women who married in their twenties revealed that family planning following marriage was a possibility. When 36-year-old Nian and her husband married she was 24 years old and they were not ready to begin a family immediately. They avoided sex during Nian’s fertile period, successfully postponing her first pregnancy by eight months. For 28-year-old Dina, her marriage occurred while she was in the midst of applying for a scholarship that required a medical examination. Had she become pregnant prior to her examination she would have effectively forfeited her opportunity to study abroad under the scholarship scheme. To prevent an unintended pregnancy Dina ensured that she and her husband were in different cities during her periods of fertility:

Belinda: Did you plan to become pregnant immediately?

Dina: No, actually we waited. Normally people try right away after marrying, right? For us we wanted to delay pregnancy because I had a medical check-up and x-ray for my scholarship. So I told my husband “I can’t get pregnant now, I’ll be ready to start trying after my check-up”.

Belinda: So how did you prevent pregnancy?

Dina: Oh *iya*, every time it was my fertile period I’d leave [laughing] … One time I went to Sumba, East Nusa Tenggara – seriously! ... Just for one week at a time, I’d be back here when I wasn’t fertile.

The narratives of both Dina and Nian reveal that their understandings of family planning included the possibility of postponing their first pregnancies to a time that suited them (and their husbands). Reproductive agency for both Nian and Dina was manifested in their ability to negotiate delaying their first pregnancy through open communication with their husbands. Another facet enabling Dina’s reproductive agency was her mobility to leave Yogyakarta, which was also critical to her and her husband avoiding the temptation to have sex during her fertile window.

However, for several other participants their reproductive agency was more limited. Twenty-three-year-old Ajeng and 21-year-old Amalia had not been able to negotiate postponing their pregnancies with their new husbands, despite their desire to do so. Ajeng became pregnant after just one month of marriage:

Ajeng: We married in April, I had my period in May, and in June I didn’t get my period… it wasn’t planned.

Belinda: Oh, you wanted to wait a bit longer?

Ajeng: Yes.

The parents of 21-year-old Amalia did not allow her and her husband to date (*pacaran*). Thus for two years before they were permitted to marry their relationship was platonic, ‘just friends’, as she describes it. Following their nuptials Amalia revealed that although she and her husband were not specifically avoiding pregnancy, she did not feel ready for children:

Amalia: After we married we just had sex normally – we weren’t trying to prevent pregnancy… I was pregnant after three months… At the time that was the intention *ya*. You’re married – of course you want to have a child *ya*.

Belinda: Your husband is quite a bit older too, right?

Amalia: Yes, he’s already in his thirties. Actually at the time I didn’t feel ready, maybe because of my age. I wanted to enjoy our marriage first, I wanted to have the experience of *pacaran*, but I got pregnant right away.

Belinda: You didn’t really have time for *pacaran*, ya?

Amalia: *Iya*, three months… alas that’s not enough time for *pacaran*!

Amalia’s narrative highlights the how personal desires can conflict with social expectations that marriage should be consummated through pregnancy as soon as possible. In order to meet this obligation, Amalia felt she had missed out on an important part of her union with her husband, and would have preferred to spend longer as a couple before starting a family. However Amalia’s ability to negotiate to defer her first pregnancy, and thus her reproductive agency, were constrained. Her reproductive agency was limited, first by her parents who would not allow a private courtship relationship. Then, by the pressure to become pregnant soon after marriage, which was further reinforced by her husband’s different priorities as a man more than ten years her senior.

### Spacing and preventing pregnancy

The duration of the postpartum ‘waiting’ or ‘seclusion’ period (*masa nifas*) was understood unanimously among women in this study as being the length of time that vaginal bleeding continued immediately following childbirth – typically 40 days. For some women contraception was not regarded as an urgent concern until after both *masa nifas* or the resumption of their menses, whereas others began using a method of contraception immediately after delivery or during *masa nifas*. In terms of the resumption of sex, nine women had abstained for one to two months postpartum; seven women had abstained for three to five months; and three women had abstained for six months or longer. Several women explained that their postpartum abstinence was rooted in Javanese cultural beliefs pertaining to sperm tainting breastmilk through sex. One woman who was interviewed at ten weeks postpartum was abstaining, and was unsure when her intimate relationship would resume.

Ten participants were intending on having more children, while ten were not. Of the latter group, eight women were already using a fertility control method (five biomedical, three non-biomedical), Two women had not yet began using a method but their intention was to use a biomedical method. Of the participants who were planning to have more children, seven were relying predominantly on non-biomedical methods (including condoms) and three were using biomedical methods. The preferred gap between pregnancies for those intending to have more children was a minimum of two years and up to six years.

The fertility control method known as lactation amenorrhea method (LAM) was poorly understood by most participants, despite the fact that the majority had performed exclusive breastfeeding. Use of LAM is recommended for a maximum of six months postpartum only for women who are exclusively breastfeeding (defined as feeding an infant only breastmilk), and whose menstrual bleeding has not resumed [19]. Most participants who were or had exclusively breastfed did not acknowledge LAM as a method of fertility control. However one participant, 36-year-old Gita, explained her use of LAM to space her pregnancies:

I have been using natural *KB* (family planning) through breastfeeding… hopefully it works, ya. Thank God (*Alhamdulillah)* the gap between children has not been too close, three years between each.

Though they had achieved spaces of three years between their three children using LAM, Gita and her husband had relied on LAM for much longer than the recommended maximum six months – their youngest child was 13 months old. Thus Gita’s limited understanding of and extended use of LAM placed her at risk of unplanned pregnancy, potentially compromising her reproductive agency as a consequence.

When participants were asked which contraceptive methods they could safely use, the majority were unable to clearly articulate all methods readily available in Yogyakarta. As a consequence most were making decisions concerning how to control their fertility based on incomplete understandings of the contraceptive options that are legally promoted in Indonesia. Several women explicitly requested further information on postpartum family planning during interviews.

Participants’ postpartum family planning method choices were often influenced by the experiences and recommendations of their family members and friends:

My parents didn’t use *KB*. So I’ve been somewhat indoctrinated.

Aliyah, 30, using non-biomedical methods for spacing pregnancy

My sister is using the IUD too. She changes it every five years… she’s had no problems with it.

Ajeng, 23, using an IUD for spacing pregnancy

I’ve never used hormonal contraceptives… it seems like they’re not good, so it’s better not to use them. I have a friend whose breastmilk supply decreased, another became moody, then there was one who got pimples, and another who put on weight. So I don’t want to take the risk [laughs].

Harum, 28, using an IUD for spacing pregnancy

*KB* seems too risky… some friends have shared their experiences… one had an implant which disappeared within her body, it couldn’t be removed… another took the Pill which affected her hormones, her skin went dull. So I don’t think there’s a safe method aside from natural *KB.*

Susi, 26, intending to use non-biomedical methods to prevent pregnancy

Participants’ narratives revealed how the experiences of family members and friends provide them with a reference point on selected contraceptive methods. However these experiences are not impartial nor can they replace family planning counselling. Thus, when women’s family planning choices are solely or even largely influenced by the experiences of others, women are constrained in making a truly informed choice due to the partial nature of the knowledge they possess. This constraint on women’s knowledge can in turn undermine their reproductive agency.

### Family size

With the exception of one participant who revealed she would like three or four children, all were intending to have a total of two children (12 women) or three children (seven women). For some participants their desired family size was linked to the normative ideal that a complete family comprises at least one child of each sex, as emphasised by 38-year-old Mulia:

[We want] just two [children]… most important is that we already have a boy and a girl … we have a complete family with the two. If I’d had one boy and then another, my husband would probably still want a girl [laughs]… you must have a complete family.

Thus the prior pregnancies of several participants had been for the purpose of achieving the ‘complete family’, comprising at least one boy and one girl. Thirty-three-year-old Ida had first had twin sons and her second pregnancy was an attempt to complete the family with a daughter:

God willing this is enough for now… actually I was hoping the last one would be a girl… [laughs].

When participants were asked about their desired family size several revealed there was a discrepancy between their preference and their husband’s, with their husbands wanting larger families. This was illustrated by 33-year-old Maria:

For me three is enough, but my husband would like to have six children.

Amalia’s husband had a fatalistic outlook on their family size, whereas she had a clear limit:

My husband wants as many children as God gives us, but privately I do have a target of just three children.

Amalia’s narrative also revealed the couple’s lack of agreement concerning the timing of subsequent pregnancies: she wanted a gap of at least five years, while her husband wanted a much shorter gap. Amalia had been able to delay her next pregnancy because she intended to breastfeed her daughter for two years and perceived breastfeeding as incompatible with pregnancy:

I want a gap of five or six years, but he wants two years – the other day he said just a one year gap would be fine–wow (*aduh*)! But we can’t, I won’t be able to breastfeed her for two years… if you’re pregnant you’re not allowed to breastfeed, *ya*? ... Maybe you’ve heard this already, if a woman is pregnant she can’t produce breastmilk… and if she does breastfeed it automatically brings on contractions *ya*.

Thus through Amalia’s understandings of combining breastfeeding and pregnancy, though not necessarily accurate from a biomedical perspective, she influenced her husband to allow a longer space between pregnancies. This would also potentially help her to achieve the smaller family size that she preferred.

### Accessing postpartum family planning

Participants unanimously described the term family planning (*KB*) as synonymous with the GoI’s national family planning program. Participants perceived family planning to be centred on limiting family size, primarily through the use of biomedical contraception to achieve the government-driven agenda of fertility control. The alternative to biomedical contraception was referred to by participants as natural family planning or *KB alami*, a mode of fertility control managed by participants and their husbands independent of biomedical consultation and intervention. Here our focus is on the experiences of women who had accessed postpartum family planning via the health system. Thirteen participants had engaged only with the private health sector (hospitals, maternal health clinics, and midwife clinics) for their reproductive health care, four participants has accessed care through both the private and public sectors, and three had engaged only with the public sector.

Both Ajeng and Ida had accessed family planning via the public health sector. Their experiences reveal the limits placed on their reproductive agency in their interactions with public sector family planning providers. Though Ajeng had come to terms with using the IUD, she had initially refused it:

It was inserted right away. At the time I refused, but the doctor told me “you have to have it, its mandatory”… I actually didn’t realise at the time it had been inserted because I was still under anaesthetic from the caesarean.

Ajeng’s narrative highlights her clear lack of choice at an extremely vulnerable time, and could be constituted as assault. She lacked the ability to decide when to begin using the IUD, and because she had been anesthetised for her C-section delivery she was unaware at the time that she was having the IUD inserted. It was evident that Ajeng’s right to give or refuse informed consent had not been respected.

For Ida, who also sought care in the public system, her ability to use her preferred postpartum contraceptive method was delayed, stemming from information she received from a midwife at the primary health clinic:

Ida: It’s safe to use *KB* after *masa nifas*. Normally 40 days after delivery you can begin using *KB.* But while I was breastfeeding I was not allowed to use IUD or injectable contraceptives (*suntik*).

Belinda: Why couldn’t you use IUD or *suntik* at that time?

Ida: Because after giving birth, our menstruation has not returned, right? So, in between the delivery and return of menstruation you can use POP (*KB pil menyusui*) – the pill for breastfeeding women. If you want to change methods you have to wait for menstruation first… my menstruation began after nine months.

Belinda: Nine months, and then you began using an IUD?

Ida: Yes, that’s right, after menstruation that’s what the midwife at the *puskesmas* (primary health clinic) told me, if you want to change *KB* methods, you have to wait for your menstruation and after that, *ya*, I began using an IUD.

Ida’s narrative illuminates how her understandings of postpartum family planning had been shaped by misinformation provided by a family planning provider that was assumed to be accurate. This compelled Ida to delay using the IUD, and for the first nine months following delivery she relied on the POP. Given that the POP has to be taken at exactly the same time each day to be effective, compared with the IUD (which once inserted is effective immediately) this potentially increased the chance of Ida experiencing unintended pregnancy. In this way, Ida’s reproductive agency was constrained, as her intention to use the method she wished to use, when she wanted to use it, was undermined by directives of her family planning provider.

Thirty-seven-year-old Prima had an IUD inserted postpartum immediately following her vaginal delivery by a public family planning provider. Prima’s IUD was removed soon after insertion due to postpartum bleeding and she had not had another inserted, nor begun using another contraceptive method. She was unsure which method she would use in the future and expressed concerns that family planning providers did not share adequate information during family planning counselling, despite her clear desire to know more:

… Maybe it would be different if I was socialised again, I would have a better understanding of the side effects associated with *KB*. The government has to be more transparent … whether the side effect is drowsiness, increased heartbeat or changes to the normal menstrual cycle… or if the hormones or ingredients used can lead to illness or cancer in people who are already susceptible… Health workers and doctors know more, and they need to be more open in their delivery of information, so we know the bad, the good, and the risks, so we can make the right choice.

The narrative of 35-year-old Bunga, who accessed family planning via a private specialist doctor, provides a contrast to the experiences of Ajeng, Ida and Prima. It is also consistent with the experiences of other participants who had accessed family planning or received counselling on contraceptive methods from private sector providers. Bunga’s prior pregnancy resulted from an IUD failure and was thus unplanned. She had opted for sterilisation to prevent future pregnancies:

The sterilisation operation was directly after the Caesarean. From early during the pregnancy the doctor had heard my medical history… they told us what the options were. I was fearful of the IUD, I didn’t want to use the Pill because I don’t want more children. Sterilisation was the best option my husband and I agreed, because the doctor told us it was the safest.

It was evident from Bunga’s narrative that she had received comprehensive family counselling, her doctor had informed her of a range of options, and she had the opportunity to consider the options before giving birth. In this way Bunga’s family planning provider supported her reproductive agency by assisting her to make an informed choice.

## Discussion

Improving reproductive health has been a persistent challenge for Indonesia and there is great potential for postpartum family planning to contribute to that end [10–13]. Yet exploration of the family planning perceptions and choices of Indonesian women, specifically during the postpartum phase, has previously been lacking. The narratives of women who participated in our study reflect the socially embedded nature of postpartum family planning understandings and decision making in Indonesia, which aligns with recent research in other lower income settings [24–28, 30]. We have demonstrated how in the Indonesian context normative social expectations concerning women’s reproductive roles and fertility, the experiences of family members and friends, conjugal negotiations, and interactions with the health system shape the way postpartum women understand and make choices about family planning. Our analysis extended to considering how women’s relationships, and socially embedded understandings of reproduction and fertility, influence their reproductive agency. Specifically, we have highlighted how the reproductive agency of women in our study manifested in their family planning decisions. Our findings also reveal the ways in which women’s social interactions and societal norms have the effect of shaping their family planning understandings and choices in ways that sometimes constrain, rather than enhance, their reproductive agency.

Participants’ desire to begin a family soon after marriage was unanimous, and was particularly pressing for women such as Nurul who wed at a later age. Women’s narratives illustrated the prevailing social expectation that a successful union involves reproduction. This is due to the primacy afforded to motherhood, perceived to enable women to fulfil their destiny (*kodrat wanita*), and its central in the social construction of idealised womanhood [39, 43, 55]. These understandings compelled Amalia and Ajeng to become pregnant soon after marrying, despite their desire to delay reproduction. Raman and colleagues [27] reported similar findings in their research with postpartum women in South India, concluding that individual choices concerning reproduction are limited. Yet the experiences of several women in our study, Nian and Dina, revealed that it is possible within some marriages to negotiate and achieve postponed reproduction, albeit through the use of non-biomedical methods. For our participants decision-making concerning family planning after marriage was influenced by these prevailing societal norms, while the actual negotiations occurred within their marital relationships. In the Indonesian context the nuclear family remains the primary locus in which reproductive decisions are made, differing from South Asian kinship systems [26, 27].

Given that contraceptive use is not normative before reproduction in Indonesia, it follows that family planning is contemplated by women and couples for the first time during or after the postpartum period. Most of the women in our study, particularly first time mothers or those who had never used biomedical contraception, had limited understandings of postpartum contraception. Despite the majority of women in our study undertaking exclusive breastfeeding, their understanding of LAM was also limited, as has been identified in other recent research [56–58]. Moreover the conclusion of *masa nifas* was not perceived by women to be an especially urgent time to begin using contraception, even though many were at risk of unintended pregnancy. Thus our findings highlight how women’s priorities during the postpartum phase deviate from the global public health agenda that promotes the use of family planning during the postpartum period to prevent unintended pregnancy and achieve safe spacing between pregnancies.

It was commonplace for the family planning understandings and experiences of others to shape those of the women in our study. Mbekenga and colleagues [31] reported similar findings in a qualitative study of first time mothers in Tanzania (*n* = 10). Their participants were more reliant on the support and advice they received from their family members and friends than they were on the formal information they received from health workers [31]. Another recent study of postpartum Indonesian women in Klaten, Central Java (*n* = 19) found that women had poor health literacy concerning postnatal care [59]. This limited health literacy, combined with intergenerational norms and myths, and the social power of husbands, parents and in-laws, were found to influence women’s lack of engagement in postpartum healthcare [59]. Considering that understandings of family planning were limited for the women in our study, the influence of others within their interpersonal circles is a concern, as it is highly likely that their understandings are also incomplete. This may perpetuate incomplete understandings of postpartum family planning, and in turn limit the scope of contraceptive options to those that have been tried and tested (with positive results) by others.

The ‘prosperous family’ (*keluarga sejahtera)* ideal, promulgated by the GoI via the national family planning program, promotes small nuclear families [60, 61]. The program’s long-standing slogan ‘*dua anak cukup*’ (two children is enough) – and, more recently, ‘*dua anak lebih baik*’ (two children is better) – is firmly embedded in the Indonesian psyche [9]. The narratives of women in our study revealed that their desired family size was aligned with this small family model, but that it was not uncommon for their husbands to want larger families. Consequently women’s decisions concerning family size were the subject of ongoing spousal negotiation, as per other reproductive decisions.

Our findings also revealed compromised quality of care when family planning was accessed via the public sector (see [62]). This manifested in the constraint of women’s choice of methods due to poor technical competence, as was experienced by Ida; or methods being forced upon women and without their consent, as revealed by Ajeng’s narrative. These accounts are reminiscent of the substandard quality of care during IUD and contraceptive implant ‘safaris’ documented in Indonesia during the 1990s [63–65]. Prima explicitly called for clearer and more comprehensive information from family planning providers. Similar challenges concerning the transfer of reproductive health information to patients within the Indonesian health system have been established by Bennett [40] and Bennett and colleagues [43, 66]. Thus our findings further emphasise the potential for health system strengthening in the realm of family planning quality of care to assist Indonesian women to realise their reproductive agency.

### Recommendations

Three clear recommendations for supporting women’s reproductive health outcomes and quality of care as it pertains to postpartum family planning flow from our findings. First, there is a need for the GoI to consider the timing of family planning education for both women and men. This is especially important for women, to assist them make more informed postpartum family planning choices, to understand their rights, and to help them negotiate their reproductive desires within their marriages. The postpartum period – particularly in the initial days and weeks following a delivery – is typically a vulnerable time for women, physically and emotionally. Women would benefit from a stronger knowledge base from which to make their family planning decisions, however the postpartum period itself is not the ideal time to first be presenting this information to women and couples. We suggest that family planning education needs to begin much earlier – preferably before marriage, to assist couples to negotiate their priorities at the outset of their relationship. Ideally this education would begin within a comprehensive sexuality education (CSE) curriculum and continue later in the context of pre-marriage counselling sessions (*konseling pranikah*) which are becoming increasingly popular.^5^ Embedding postpartum family planning education and counselling within routine antenatal care would also provide another window of opportunity to educate women about the fertility control options available, giving them an opportunity to consider the various methods well in advance. The second recommendation emerging from this study relates to the content of family planning education, which we believe should not be limited to information about biomedical contraception, but should adopt a wider framework as per the WHO definition of family planning [67], encompassing planning family size, pregnancy spacing and timing, contraception, including postpartum fertility control and the correct use of LAM for breastfeeding women, and infertility treatment. Our final recommendation relates to the substantial scope to improve the patient education skills of family planning providers, informed by the gaps in knowledge among participants identified in this study, which would have the flow-on effect of improving the quality of family planning counselling they provide. It is especially pertinent for family planning providers to learn the current protocols on women’s eligibility for postpartum family planning methods, and for their knowledge to be continually updated as these protocols evolve.

### Study limitations

A limitation of our study was that we sought to explore in-depth the family planning understandings and choices of postpartum women in urban Yogyakarta, thus our results are not generaliseable beyond this population. Yogyakarta is a unique setting in that it is regarded as Indonesia’s higher education city and thus a much greater proportion of the population has a high level of education compared with other provinces across the archipelago. Given that family planning decisions are typically made by women in consultation with their husbands, and the patriarchal nature of gender relations in the Indonesian context, it may be pertinent for a future study to consider family planning understandings and decisions from the perspective of men. However our participants were highly educated, largely from middle class backgrounds, and typically older when they married than the national average. Thus we conceived they had a reasonable basis from which to negotiate with their husbands in comparison with poorer, younger and less educated women in which the gendered power imbalance between women and men tends to be (but is not always) greater [40, 68–70]. Moreover, while some participants’ husbands and other family members were present in the home during IDIs, we did not specifically interview them. The presence of husbands and other family members may have constrained what participants were willing to share in some cases.

## Conclusions

Our findings reveal the ways in which Indonesian women’s reproductive agency is undermined at three distinct junctures. First, through their incomplete understanding of postpartum family planning; second, by skewed information they receive in their interactions with others, including family planning providers; and third, through societal expectations concerning their fertility and reproduction. This necessitated our analysis of the relational context in which women’s decisions concerning postpartum family planning are embedded. Our findings demonstrate the need for the provision of timely and comprehensive family planning education to women, to assist them to make more informed choices, enhancing their reproductive agency. Ideally both women and men need to be privy to this education because ultimately decisions concerning contraception, family size and pregnancy spacing are made within the marital unit. Our findings also revealed that family planning counselling and the patient education skills of family planning providers have much scope for improvement to enhance quality of care provided to women and couples, which would further support women’s reproductive agency.

## Abbreviations

AIMI: Indonesian Breastfeeding Mothers’ Association *(Asosiasi Ibu Menyusui Indonesia)*
CSE: Comprehensive sexuality education
GoI: Government of Indonesia
IDHS: Indonesian Demographic and Health Survey
IDI: In-depth interview
IUD: Intrauterine device
KB: Family planning *(keluarga berencana)*
LAM: Lactation amenorrhea method
MMR: Maternal mortality ratio
POP: Progestogen-only pill
TFR: Total fertility rate
WHO: World Health Organization

## Footnotes

1 In the 2012 Indonesian Demographic and Health Survey unmarried women were for the first time included in the calculation of MMR; which raised the MMR from 220 to 359 [3]. Unmarried women in Indonesia remain unable to legally access family planning services and may only have access to safe and legal abortion services in case of rape.

2 Interviews with several participants were interspersed with some English and Javanese at the participants’ discretion.

3 As mentioned above, one participant referred by snowballing chose not to disclose her contact details to BRS and the interview was set up via her neighbour (also a participant).

4 It was determined that literacy would not be a concern for the participants sampled in this study due to their high levels of education.

5 Yet it must be noted that despite the GoI’s purported commitment to CSE, the implementation, content and quality of sexual and reproductive health education remains uneven and when it does occur, it is usually focused on the biological aspects of reproduction and promoting sexual abstinence [71–73]. A further setback to CSE occurred in late 2015 after the rejection of a request for judicial review of national education law to embed reproductive health education in the national curriculum by the constitutional court on the basis that the activist group who instigated the request has no legal standing [74]. Until a resolution has been achieved in relation to the timing of CSE, reproductive health education in Indonesia will likely remain deficient.
